# Role of hematological parameters in the diagnosis of influenza virus infection in patients with respiratory tract infection symptoms

**DOI:** 10.1002/jcla.23191

**Published:** 2020-01-04

**Authors:** Qingzhen Han, Xiaomin Wen, Lin Wang, Xiu Han, Yimin Shen, Jun Cao, Qunxin Peng, Jie Xu, Lina Zhao, Jun He, Hong Yuan

**Affiliations:** ^1^ Center of Clinical Laboratory The First Affiliated Hospital of Soochow University Suzhou China; ^2^ Department of Clinical Laboratory Shiqian People's Hospital Tongren China; ^3^ Department of Clinical Laboratory Suzhou Dushuhu Public Hospital Suzhou China

**Keywords:** hematological parameters, influenza virus infection, neutrophil‐to‐lymphocyte ratio, platelet, respiratory tract infection

## Abstract

**Background:**

The differential diagnoses of patients hospitalized for respiratory infections due to influenza virus vs other pathogens are challenging. Our study investigated whether hematological parameters such as neutrophil (N), lymphocyte (L), platelet (PLT), and neutrophil‐to‐lymphocyte ratio (NLR) contributed in diagnosing influenza virus infections and in discriminating other respiratory infections.

**Methods:**

We retrospectively analyzed the laboratory characteristics of 307 patients with respiratory infections caused by influenza/non‐influenza virus and bacteria. The diagnostic abilities of hematological indexes were evaluated in the patients compared with 100 healthy people.

**Results:**

The hematological parameters in patients with influenza virus infection were dramatically altered compared with those in the controls. Additionally, among the systemic inflammatory markers, the sensitivity of NLR for influenza detection was higher than that of N and L. PLT was significantly lower in influenza virus‐positive infection than in influenza virus‐negative infection. Moreover, when patients with influenza virus infection were cured, PLT returned to a normal level. The red blood cell (RBC) and hemoglobin (Hb) levels of influenza virus infection were higher than those of bacterial infection. Compared with traditional N and L, NLR and platelet‐to‐neutrophil (PNR) showed greater significance between influenza virus and bacterial infection (*P* < .01).

**Conclusion:**

Neutrophil‐to‐lymphocyte ratio with high sensitivity is a preferable diagnostic tool to screen influenza virus‐infected patients than N and L. PLT accounts in the differential diagnoses of respiratory infections due to influenza virus and other pathogens among patients. In addition, RBC, Hb, NLR, and PNR can significantly differentiate between influenza virus infections and bacterial infections.

## 1 INTRODUCTION

Annual seasonal influenza epidemics of variable severity result in significant morbidity and mortality worldwide.^1^ Since avian influenza was first identified in Shanghai, China, in March 2013, there have been a total of five epidemics.^2^ Patients with influenza virus mostly present with fever and cough are prone to progression to viral pneumonia. Moreover, in the event of acute respiratory distress and important organ dysfunction, the fatality rate is even higher. In addition, late diagnosis of community‐acquired influenza A virus infection is associated with a delay in ICU admission, greater possibilities of respiratory and renal failure, and higher mortality rate. Delay in diagnosis of flu is an independent variable related to death. Therefore, early diagnosis and treatment with antivirals are critical for achieving effective therapeutic outcomes.^3^

At present, molecular assays (eg, nucleic acid amplification tests and antigen tests) targeting respiratory tract specimens are recommended as critical diagnostic tests for clinical decision‐making according to influenza clinical practice guidelines in different countries.^4^, ^5^ However, these tests are limited by some technical provisions and specifications for molecular assay utilization, especially in underdeveloped areas and community hospitals. Furthermore, antigen tests have poor sensitivity to some influenza viruses.^6^, ^7^ Recently, it was reported that hematological inflammatory indexes based on blood cell analysis had an important predictive value for the prognosis of infections, cancers, and many other diseases.^8^, ^9^, ^10^ This study aimed to conduct a retrospective analysis of hematological inflammatory parameters (eg, neutrophils, lymphocytes, platelets) and blood cell count indexes, particularly the NLR, in hospitalized patients with suspected influenza. Moreover, this study aimed to validate hematological indexes as potential indicators to discriminate influenza virus infection from non‐influenza infection, which would facilitate a clear diagnosis and enable the initiation of antiviral treatment as early as possible when molecular assays for respiratory specimen tests are not performed.

## 2 MATERIALS AND METHODS

### 2.1 Study population

The present study retrospectively enrolled 307 suspected influenza virus‐infected patients with typical acute onset of respiratory symptoms (cough, rhinorrhea, and congestion), myalgia and headache with or without fever at the First Affiliated Hospital of Soochow University from January 2017 to June 2019. The diagnostic criteria for influenza virus infection included the guidelines for the diagnosis and treatment of influenza combined with positive influenza virus nucleic acid detection. Bacterial infection was confirmed by bacterial cultures. Finally, 107 patients were diagnosed with definite influenza virus infection (influenza virus positive), of which 88 had influenza A, 16 had influenza B, and 3 had combined influenza A and B (53 male and 54 female; age range: 9‐91 years; mean age: 56.54 ± 18.84 years). A total of 109 patients with respiratory symptoms were diagnosed with bacterial infection by bacterial cultures, including 33 cases of *Klebsiella pneumoniae*, 9 cases of *Pseudomonas aeruginosa*, 28 cases of *Acinetobacter baumannii,* and 39 cases of other bacterial species (79 male and 30 female; age range: 13‐92 years; mean age: 63.46 ± 18.53 years). A total of 91 patients were identified as negative controls with typical respiratory symptoms; these patients were negative for both the nucleic acid and bacterial culture results (58 male and 33 female; age range: 23‐95 years; mean age: 56.04 ± 18.53 years). In addition, 100 individuals were recruited for the control group (healthy controls) (60 male and 40 female; age range: 26‐64 years; mean age: 41.53 ± 9.88 years) (Figure 1).

**Figure 1:** Flowchart of the included patients. All patients with respiratory symptoms and without other diseases. There was no significant difference in age and sex among all enrolled people

### 2.2 Blood analysis for the determination of infection

The complete blood count was routinely examined in hospitalized patients with suspected influenza virus infection in the study. Two milliliters of peripheral blood was placed in hemogram tubes with ethylenediaminetetraacetic acid (EDTA). The blood count was determined using an automated hematology analyzer (Sysmex‐20 instrument, Sysmex). The NLR was calculated as neutrophils/lymphocytes, the PLR as platelets/lymphocytes, and the PNR as platelets/neutrophils. The viral nucleic acid of respiratory tract specimens was detected using a Viral Nucleic Acid Isolation Kit (silica‐based spin column) (BioPerfectus Technologies) and an Influenza A and B Polymerase Chain Reaction (PCR) Fluorescence Diagnostic Kit (BioPerfectus Technologies) with a Roche LightCycler 480 sequence detection system (Roche) according to the manufacturer's instructions.

### 2.3 Statistical analysis

Continuous variables are summarized as the mean ± SD (standard deviation). Student's *t* test for independent samples was used to compare continuous variables. A significance level of 0.05 was used for all statistical tests. SPSS software version 22.0 (SPSS) was used for all statistical analyses.

## 3 RESULTS

### 3.1 Comparison of diagnostic sensitivity of N, L, and NLR

The results showed that WBC, N, RDW, NLR, and PLR increased significantly in the influenza virus infection group compared with the healthy control (*P* < .01 for all), while L, RBC, Hb, PLT, and PNR decreased (*P* < .01 for all) (Table 1). Specifically, the sensitivity of NLR detection was higher than the common systemic inflammatory markers, including neutrophils and lymphocytes (Table 2). No significant differences were found between influenza virus A and B.

**Table 1:** Comparison of hematological parameters between the influenza virus infection group and the healthy control group

	Influenza virus infection (N = 107)	Healthy control (N = 100)	*P* value
WBC (10^9^/L)	8.005 ± 6.287	5.981 ± 1.175	.002**
N (10^9^/L)	6.247 ± 5.700	3.226 ± 0.913	<.001***
L (10^9^/L)	1.167 ± 1.341	2.111 ± 0.429	<.001***
RBC (10^12^/L)	3.877 ± 0.921	4.835 ± 0.445	<.001***
Hb (g/L)	116.720 ± 28.428	146.18 ± 12.977	<.001***
RDW (%)	13.628 ± 2.820	12.213 ± 0.546	<.001***
PLT (10^9^/L)	169.869 ± 93.379	229.38 ± 47.260	<.001***
NLR	8.877 ± 9.855	1.595 ± 0.507	<.001***
PNR	53.338 ± 58.693	75.406 ± 25.935	<.001***
PLR	241.042 ± 212.375	112.632 ± 30.255	<.001***

Note

Student's *t* test for independent samples was used to compare continuous variables.

Abbreviations: Hb, hemoglobin; L, lymphocyte; N, neutrophil; NLR, neutrophil‐to‐lymphocyte ratio; PLR, platelet‐to‐lymphocyte ratio; PLT, platelet; PNR, platelet‐to‐neutrophil ratio; RBC, red blood cell; RDW, red blood cell distribution width; WBC, white blood cell.

* *P* < .05.

** *P* < .01.

*** *P* < .001.

**Table 2:** Comparison of the diagnostic sensitivity for N, L, and NLR

	Influenza virus infection (N = 107)	Healthy control (N = 100)	Reference range	Sensitivity	*P* value
N (10^9^/L)	6.247 ± 5.700	3.226 ± 0.913	1.8‐6.3	37.40%	<.001***
L (10^9^/L)	1.167 ± 1.341	2.111 ± 0.429	1.1‐3.2	60.75%	<.001***
NLR	8.877 ± 9.855	1.595 ± 0.507	0.581‐2.61	70.09%	<.001***

Note

The reference range of NLR was the 95% confidence interval of NLR in the control group, *P* < .01. Student's *t* test for independent samples was used to compare continuous variables.

* *P* < .05.

** *P* < .01.

*** *P* < .001.

### 3.2 Comparison of hematological parameters between influenza virus‐positive infection and influenza virus‐negative infection

In the present paper, we found that PLT was lower in the influenza virus infection group (169.869 ± 93.379) than in the negative control group (226.209 ± 119.245) (*P* < .001), while Hb was higher (*P* < .05). Moreover, the other routine blood parameters did not differ significantly between the two groups (*P* > .05) (Table 3). In addition, L and PLT increased to normal levels concomitantly when influenza patients were completely cured (*P* < .05). Furthermore, no other hematological parameters were found to have significance with a complete cure of influenza (*P* > .05) (Table 4).

**Table 3:** Comparison of hematological parameters between influenza virus infection and negative control

	Influenza virus infection (N = 107)	Negative control (N = 91)	*P* value
WBC (10^9^/L)	8.005 ± 6.287	8.491 ± 4.725	.545
N (10^9^/L)	6.247 ± 5.700	6.538 ± 4.613	.697
L (10^9^/L)	1.167 ± 1.341	1.111 ± 0.656	.716
RBC (10^12^/L)	3.877 ± 0.921	3.671 ± 0.33	.103
Hb (g/L)	116.720 ± 28.428	109.143 ± 24.265	.047*
RDW (%)	13.628 ± 2.820	14.136 ± 3.027	.223
PLT (10^9^/L)	169.869 ± 93.379	226.209 ± 119.245	<.001***
NLR	8.877 ± 9.855	8.905 ± 9.617	.984
PNR	53.338 ± 58.693	52.994 ± 7.923	.967
PLR	241.042 ± 212.375	286.538 ± 332.511	.967

Note

Student's *t* test for independent samples was used to compare continuous variables.

* *P* < .05.

** *P* < .01.

*** *P* < .001.

**Table 4:** Comparison of hematological parameters before and after treatments

	Pretreatment (N = 64)	Posttreatment (N = 64)	*P* value
WBC (10^9^/L)	8.490 ± 5.567	8.519 ± 4.744	.975
N (10^9^/L)	6.858 ± 5.392	6.444 ± 4.561	.640
L (10^9^/L)	0.996 ± 0.606	1.365 ± 0.765	.003**
RBC (10^12^/L)	4.054 ± 0.794	3.896 ± 0.738	.245
Hb (g/L)	122.594 ± 23.525	117.016 ± 22.424	.172
RDW (%)	13.775 ± 3.137	15.221 ± 12.490	.370
PLT (10^9^/L)	188.5 ± 89.146	232 ± 103.899	.012*
NLR	10.179 ± 11.003	7.228 ± 11.290	.137
PNR	48.437 ± 44.892	51.849 ± 36.353	.637
PLR	255.983 ± 180.771	212.560 ± 126.046	.117
WBC	8.490 ± 5.567	8.519 ± 4.744	.975

Note

Student's *t* test for independent samples was used to compare continuous variables.

* *P* < .05.

** *P* < .01.

*** *P* < .001.

### 3.3 The differential sensitivity of hematological parameters between influenza virus infection and bacterial infection

Compared with bacterial infection, RBC, Hb, and PNR markedly increased in influenza virus infection, while WBC, RDW, neutrophils, and NLR decreased (Table 5).

**Table 5:** Comparison of hematological parameters between influenza virus infection and bacterial infection

	Influenza virus infection (N = 107)	Bacterial infection (N = 109)	*P* value
WBC (10^9^/L)	8.005 ± 6.287	9.792 ± 4.525	.039*
N (10^9^/L)	6.247 ± 5.700	8.058 ± 4.679	.027*
L (10^9^/L)	1.167 ± 1.341	0.998 ± 1.076	.373
RBC (10^12^/L)	3.877 ± 0.921	3.453 ± 0.837	.002**
Hb (g/L)	116.720 ± 28.428	105.625 ± 24.964	.008**
RDW (%)	13.628 ± 2.820	14.764 ± 2.442	.006**
PLT (10^9^/L)	169.869 ± 93.379	146.653 ± 79.849	.086
NLR	8.877 ± 9.855	18.933 ± 38.447	.009**
PNR	53.338 ± 58.693	26.344 ± 22.243	<.001***
PLR	241.042 ± 212.375	282.231 ± 335.472	.283

Note

Student's *t* test for independent samples was used to compare continuous variables.

* *P* < .05.

** *P* < .01.

*** *P* < .001.

## 4 DISCUSSION

A late diagnosis of influenza virus infection is associated with greater possibilities of respiratory and renal failure and a higher mortality rate.^3^ Due to shared routes of transmission, coinfection with influenza virus and bacteria has become common among individuals, making it even more complicated to confirm influenza virus infection and choose accurate treatments. As such, we demonstrated the relationships between laboratory parameters and influenza virus infections, bacterial infections and non‐influenza virus infections.

Blood cell count analysis is a simple, effective, and rapid laboratory diagnostic basis for evaluating infectious inflammatory responses.^11^ The influenza virus‐infected patients analyzed in this paper were mainly elderly people. Additionally, elderly people were mainly involved as the controls in this study. Therefore, the age and sex distribution of the selected controls were as close as possible to those of the influenza virus‐infected group. The results showed that routine blood indicators were independent of age and sex, consistent with the findings of previous literature reports.^12^ This study found that many hematological parameters changed significantly due to influenza virus infection, such as PLT, WBC, RBC, Hb, and RDW. Influenza virus infection induced a relatively increased N count and a relatively decreased L count, which was different from the changes caused by other common viruses such as adenovirus, respiratory syncytial virus, EB virus, human herpes virus type 6, and enterovirus.^13^, ^14^ In addition, NLR was as a more sensitive parameter for influenza virus infection than the other cell count parameters in our study, which was consistent with reports on many other diseases, such as lung cancer and swine flu.^8^, ^15^, ^16^, ^17^, ^18^ A hemogram is a basic investigation performed in all admitted patients (including patients with respiratory tract infection), and NLR can be easily calculated from the results. Previous studies have independently assessed the clinical significance of these blood markers in various patients, specifically in those with malignancies. Here, we evaluated the early predictive value of NLR in influenza virus infection. Additionally, no significant difference in hematological parameters was found between different subtypes of influenza virus A (20 H1N1, 9H7N9, and 10 H3), but further elaboration is needed in more cases.

Among patients with typical symptoms of respiratory influenza infection, only approximately 40% were truly infected by influenza virus during its seasonal peak based on the results of nucleic acid detection, and this percentage was much lower during the non‐epidemic season of influenza.^19^ The differential diagnosis of influenza virus from other microbial infections based only on clinical symptoms before performing the nucleic acid test is very challenging. In our retrospective analysis of the hematological parameters of suspected influenza patients, PLT count was significantly lower (169.869 ± 93.379) in influenza virus‐positive patients than in negative controls (226.209 ± 119.245) (*P* < .001), suggesting that decreased PLT counts could differentiate influenza virus infections from others. Furthermore, PLT count returned to a normal level concomitantly while influenza patients were completely cured, indicating that PLT count had a high correlation and specificity in influenza laboratory diagnosis. This was the first study to present real laboratory data to confirm other reports on the mechanism of platelet inhibition induced by influenza virus. It has been reported that influenza virus could induce uncontrolled platelet activation to fuel a harmful inflammatory response in the respiratory tract.^20^, ^21^, ^22^, ^23^ We hypothesized that such excessive activation of platelets by influenza virus may lead to a markedly decreased platelet count compared with other respiratory tract infections. Nevertheless, the detailed mechanism can be complex and further studies are warranted to confirm these associations.

In addition, our data demonstrated that RBC, Hb, and PNR were higher in influenza virus infection than in bacterial infection. They were differential diagnostic indicators for infection caused by influenza virus vs bacteria. At present, it is well known that influenza hemagglutinin readily binds to sialic acid receptors on the membranes of red blood cells, causing red blood cells to clump together or agglutinate.^24^ Some bacterial infections cause intravascular hemolysis leading to sepsis, which reduces the red blood cell count^25^ and may be why bacterial infections cause more significant reduction in red blood cells.

In conclusion, NLR was found to have a high sensitivity in detecting influenza virus infection. PLT count had a high correlation and specificity to preliminarily discriminate influenza virus infection from suspected influenza virus infection. In addition, RBC, Hb, NLR, and PNR showed some diagnostic value for differentiating between influenza virus infection and bacterial infection. In summary, some hematological indexes (eg, PLT, NLR, RBC, and Hb) as simple early laboratory indicators have promising value in the diagnosis of influenza virus infection. Further investigation of the reference ranges of hematological parameters based on influenza virus infection and individual physiological levels is warranted.

## AUTHORS' CONTRIBUTIONS

Jun He, Qingzhen Han, and HongYuan designed the study and revised the manuscript. Xiaomin Wen, Lin Wang, and Xiu Han performed the experiments, analyzed the data, and wrote the article. Yimin Shen, Jun Cao, Jie Xu, Lina Zhao, and Qunxin Peng contributed to the experimental work and the collection of patients’ characteristics. All authors read and approved the final manuscript.
